The article "High-Dose-Rate Intracavitary Brachytherapy Under Conscious Sedation a Viable Practical Alternative to Spinal Anaesthesia in Carcinoma Cervix: A Retrospective Study in a Tertiary Care Centre in Eastern India" was published in 2021. Journal: Cureus.

# High-Dose-Rate Intracavitary Brachytherapy Under Conscious Sedation a Viable Practical Alternative to Spinal Anaesthesia in Carcinoma Cervix: A Retrospective Study in a Tertiary Care Centre in Eastern India

**DOI:** 10.7759/cureus.20063

**Published:** 2021-11-30

**Authors:** Bikash Ranjan Mahapatra, Bijay K Barik, Anupam Muraleedharan, Avinash Badajena, Adhar Amritt, Satyabrata Kanungo, Ashutosh Pattanaik, Minakshi Mishra, Sovan S Dhar, Sandip K Barik, Saroj Kumar Das Majumdar, Dillip Kumar Parida

**Affiliations:** 1 Radiation Oncology, All India Institute of Medical Sciences, Bhubaneswar, IND; 2 Medical Physics, All India Institute of Medical Sciences, Bhubaneswar, IND

**Keywords:** dosimetry, conscious sedation, spinal anaesthesia, uterine cervical cancer, intracavitary brachytherapy

## Abstract

Introduction

Intracavitary brachytherapy (ICBT) is an integral component in the management of locally advanced cervical cancer. Spinal anaesthesia is the preferred mode of pain management during brachytherapy procedures. In high volume, resource constraint settings, it is difficult to provide spinal anaesthesia to all patients. This study attempts dosimetric comparison of high-dose-rate ICBT with spinal anaesthesia to that under conscious sedation to find out whether brachytherapy under conscious sedation is comparable with spinal anaesthesia.

Methods

Retrospective data of total of 56 cervical cancer patients who received ICBT after completion of external beam radiotherapy (EBRT) were collected. Among these 56 patients, 28 patients received brachytherapy under spinal anaesthesia (SA group) and the rest under conscious sedation (CS group). Brachytherapy dose was 7 Gray per fraction weekly for three weeks. Thus, 84 brachytherapy plans of each group were analysed with respect to doses received by points A, B, P and Organs at Risk.

Results

The mean doses received by points A, B and P were comparable in SA and CS groups (p-value >0.05). Similarly, the mean doses received by Organs at Risk (rectum, urinary bladder, and sigmoid colon) were also comparable in both the groups (p-value>0.05).

Conclusion

ICBT under CS is dosimetrically non-inferior to SA, which makes it an alternative option.

## Introduction

Cervical cancer is the second most common gynaecological cancer and the fourth most common malignancy worldwide with an annual incidence of 6.04 lakhs cases and 3.42 lakhs deaths [1]. It is more common in countries with less access to screening especially in developing and underdeveloped regions of the world. In India, cervical cancer is the third most common malignancy considering both sexes. It is also the second most common malignancy in females after breast cancer. In India, the annual incidence of cervical cancer is 124,000 cases and 77,348 deaths. Five-year prevalence is 42.8 per 100,000 population representing the second most prevalent cancer after breast cancer for both sexes [2].

The article "High-Dose-Rate Intracavitary Brachytherapy Under Conscious Sedation a Viable Practical Alternative to Spinal Anaesthesia in Carcinoma Cervix: A Retrospective Study in a Tertiary Care Centre in Eastern India" was published in 2021. Journal: Cureus.

For early-stage cervical cancer, either concurrent chemoradiation with intracavitary brachytherapy (ICBT), radical brachytherapy or surgery is recommended [3,4]. The decision regarding which modality to choose depends on disease extension, need for preservation of fertility, patient’s preference, presence of comorbidities, and access to radiotherapy facilities.

In locally advanced cervical cancer (Stages IIB to IVA) and stage IB3 [5] concurrent chemoradiation followed by ICBT is considered the standard of treatment [6-11].

ICBT is an integral part of the treatment of cervical cancer by radiotherapy because the tumoricidal dose cannot be delivered by external beam radiotherapy (EBRT) alone due to the presence of critical structures [12,13]. It is a highly conformal mode of treatment that delivers a higher dose to the cervix, uterus, parametrium, and part of the vagina with relative sparing of the surrounding critical organs. As ICBT is an invasive procedure, it needs pain management. There are various forms of pain management including general anaesthesia (GA), spinal anaesthesia (SA), intravenous conscious sedation (CS), paracervical block and oral pain management [14].

In spinal anaesthesia, patients need to undergo pre-anaesthesia clearance (PAC) unlike for conscious sedation. Post procedure, patients also require prolonged observation in view of anticipated complications. On the other hand, conscious sedation is associated with very minimal complications.

For an optimal brachytherapy procedure, muscle relaxation and patient comfort is of paramount importance. Inadequacy of either will lead to sub-optimal applicator placement as well as dose distribution. In this context, brachytherapy under GA or SA is assumed to be near perfect to achieve this goal albeit inherent complications [15]. In a resource constraint, high burden setting like many of the East Asian as well as African countries, providing GA/SA to all the patients would be of big challenge. In this context, ICBT procedure under CS appears to be an alternative.

With SA, there is better perineal muscle relaxation, so more vaginal packing is possible which is assumed to reduce dose to critical structures in comparison to that of CS. In this study, we are trying to compare the dosimetry of plans done in SA and CS and to find out whether plans in conscious sedation is dosimetrically comparable to those made under spinal anaesthesia.

## Materials and methods

High-dose-rate intracavitary brachytherapy (HDR-ICBT) was started in our centre by the end of the year 2018. Anaesthesia support for the procedure was allotted only for a single day in a week due to the shortage of manpower. Therefore, it was not possible to accommodate all patients in a single operation theatre (OT) day. Due to this reason, brachytherapy was done under CS for the rest of the week.

The article "High-Dose-Rate Intracavitary Brachytherapy Under Conscious Sedation a Viable Practical Alternative to Spinal Anaesthesia in Carcinoma Cervix: A Retrospective Study in a Tertiary Care Centre in Eastern India" was published in 2021. Journal: Cureus.

This retrospective study is intended to analyse the patients treated in our institute from January 2019 to August 2021. All the patients had received EBRT dose of 50 Gray in 25 fractions, 5 fractions per week with a concurrent weekly Inj. Cisplatin 40 mg/m^2^. After EBRT, patients were clinically assessed for ICBT and treated for a dose of 7 Gray to point A per fraction, weekly, for 3 weeks. The total treatment duration was eight weeks from the start of EBRT. The total number of patients in both the groups (SA and CS) was 28 each with a total of 84 fractions of HDR-ICBT sessions in each group.

Patient preparation for ICBT

All patients were advised for CBC, RFT, PT-INR, aPTT, viral markers (HIV, HBsAg, Anti HCV). Chest X-Ray, ECG, and 2D Echocardiography were advised specifically for those patients who were planned for the procedure under SA. In addition, patients in the SA group had to undergo Pre-Anaesthesia Clearance at the Department of Anaesthesia and Critical Care. One day prior to ICBT, in-hospital admission was done. Shaving from the umbilicus to mid-thigh was done. Bowel preparation was done by gastrointestinal lavage using 137.15 grams Polyethylene glycol powder in one litre of water which is drank over a period of two to three hours, the night prior to the procedure. Patients were kept in empty stomach from midnight. Additionally, proctoclysis enema was given three hours prior to the procedure. Then patients were shifted to the Brachytherapy patient waiting room. Informed consent was taken after explaining the procedure and its side effects. After monitoring of vital signs and reviewing pre-anaesthesia clearance (as the case may be) patients were transferred to brachytherapy OT.

Patients in the SA group received Inj. Ondansetron 8 mg IV as premedication. Agent used for SA was 2- 2.5 ml Inj. Bupivacaine heavy (5 mg/ml) depending on build of the patient and duration of procedure along with Inj. Fentanyl 25 mcg.

On the other hand, patients in the CS group received Inj. Promethazine 25 mg and Inj. Tramadol 50 mg as intravenous infusion, 30 minutes prior to the procedure. Modified Observer’s Assessment of Sedation Scale (MOASS) is used to measure the depth of sedation. 2% lignocaine spray was used locally for analgesia [16]. Prior to sedation, Inj. Ondansetron 8 mg and Inj. Pantoprazole 40 mg were given as premedication.

The article "High-Dose-Rate Intracavitary Brachytherapy Under Conscious Sedation a Viable Practical Alternative to Spinal Anaesthesia in Carcinoma Cervix: A Retrospective Study in a Tertiary Care Centre in Eastern India" was published in 2021. Journal: Cureus.

After achieving the desired level of anaesthesia/sedation, patients were taken up for ICBT application. Vital signs were monitored throughout the procedure. In the CS group, MOASS score of 3 was considered adequate. Patients were then kept in lithotomy position and the perineum was then painted with 0.5 % povidone iodine solution along with Cetrimide and Chlorhexidine gluconate solution (Savlon) followed by draping with sterile drapes. A Foley catheter was inserted and inflated with 7 cc distilled water.

Applicator selection and insertion

Per vaginal examination was done to assess the position of cervix, residual disease, negotiability of cervical os and vaginal space. Then bimanual examination was done to assess the position of the uterus (anteverted or retroverted). Per speculum examination was done for better visualisation. 2% lignocaine spray was applied in the CS group for local anaesthesia. Serial dilation of cervix was done with Hegar’s dilator. Intrauterine length was measured with a uterine sound. A modified Fletcher suit applicator was used. The appropriate size of intrauterine tandem was inserted. Then the appropriate size of ovoids were inserted into bilateral fornices which would snugly fit. Intrauterine tandem and ovoids were fixed. Roller gauze soaked in 0.5 % povidone-iodine and 2 % lignocaine jelly was used for vaginal packing. Adequate vaginal packing was done to increase the distances between applicator and surrounding structures (bladder and rectum). T band was used to hold the applicator set in a fixed position.

CT simulation and contouring of organs at risk

The patient was then transported to CT simulator (GE & Optima CT 580) with due care given not to distort the applicator position. Non-contrast CT simulation was done, and the images transferred to Oncentra Brachytherapy Planning System (V4.6.01). Organs at risk (bladder, rectum and sigmoid colon) were contoured as per RTOG guidelines [17].

Planning

CT data of the patient was then imported to Oncentra Brachytherapy Planning System (V4.6.01). On the CT images, catheter reconstruction was done and reference points such as point A, point B and pelvic wall point (point P) were created (Figure 1) [18,19].

**Figure 1:** Isodose lines and points A, B and P.

At each fraction, a total dose of 7Gy was prescribed to point A (Figure 2).

**Figure 2:** Reconstructed catheters with 7 Gy isodose volume and organs at risk.

Dose colour wash and isodose lines were examined to ensure that dose received by point A is adequate. The doses received by other reference points (points B and P) as percentages of point A dose were also evaluated. Along with that, volumetric dose evaluation for organs at risk (D0.1cc and D2cc of bladder, rectum and sigmoid as percentages of point A dose) were done from dose-volume histogram (DVH) (Figure 3) [19,20].

The article "High-Dose-Rate Intracavitary Brachytherapy Under Conscious Sedation a Viable Practical Alternative to Spinal Anaesthesia in Carcinoma Cervix: A Retrospective Study in a Tertiary Care Centre in Eastern India" was published in 2021. Journal: Cureus.

**Figure 3:** Dose-volume histogram showing D2cc to organs at risk. D2cc, the minimum dose received by 2cc volume of the organs at risk.

Treatment delivery

The patients were transported to treatment room and channels were connected between HDR unit and the applicators. At our centre, we have High Dose Rate Remote Afterloading Brachytherapy machine (Nucletron & microSelectron HDR V3) with Iridium-192 as the source. Treatment was delivered with vital signs being monitored throughout the procedure from the console.

Removal of applicator

Channels, vaginal packings and applicators were removed sequentially. Then vaginal examination was done to assess for active bleeding. If active bleeding was there, pressure packing was applied.

Assessment of pain during procedure

After completion of ICBT treatment, patients were asked about the degree of pain they felt during the procedure. Visual analogue scale (VAS) was used as a tool to record the same.

## Results

The number of patients in each group (CS and SA) were 28. All patients underwent three sessions of ICBT after completion of EBRT. EBRT dose (50 Gray in 25 fractions) as well as ICBT dose (7 Gray per fraction for three sessions) were uniform for both groups. In total, 168 ICBT plans were taken up for statistical analysis which was done by SPSS Version 21.0. The unpaired t-test was applied to compare the means between the groups.

The most common age group in SA group was 60 to 69 years (46.4%) while that for CS group was 50 to 59 years (39.3%). The ages of the patients ranged from 31 to 76 years in the SA group while it was 35 to 76 years in CS group. The most common stage in which the patients presented was stage III in SA group and stage II in CS group. Squamous cell carcinoma was the predominant histology irrespective of the groups (Table 1).

**Table 1:** Baseline characteristics between two groups. FIGO: International Federation of Gynecology and Obstetrics; EBRT: external beam radiotherapy; ICBT: intracavitary brachytherapy; SA: spinal anaesthesia; CS: conscious sedation.

Group		SA	CS
Number of patients		28	28
Number of ICBT applications		84	84
Age group of patients (in years)	30-39	3	2
	40-49	4	7
	50-59	7	11
	60-69	13	5
	70-79	1	3
FIGO stage	Stage II	12	16
	Stage III	15	11
	Stage IV	1	1
Histopathology	Squamous cell carcinoma	27	24
	Adenocarcinoma	1	1
	Adenosquamous carcinoma	0	3
EBRT Dose (in Gray)		50	50
ICBT Dose per fraction (in Gray)		7	7

The mean calculated doses, to points A, B, P and the Organs at Risk, received by the two groups (SA and CS) were comparable (Tables 2, 3). 

The article "High-Dose-Rate Intracavitary Brachytherapy Under Conscious Sedation a Viable Practical Alternative to Spinal Anaesthesia in Carcinoma Cervix: A Retrospective Study in a Tertiary Care Centre in Eastern India" was published in 2021. Journal: Cureus.

**Table 2:** Doses received by points A, B and P. SA: spinal anaesthesia; CS: conscious sedation.

Dose (% of Point A)		SA	CS	p-value
Left	Point A	99.53	99.63	0.77
	Point B	29.98	27.87	0.25
	Point P	20.37	20.18	0.50
Right	Point A	99.75	99.59	0.68
	Point B	30.02	28.23	0.36
	Point P	20.26	20.45	0.54

**Table 3:** Doses received by organs at risk. SA: spinal anaesthesia; CS: conscious sedation.

Dose to organs at risk (% of Point A)		SA	CS	p-value
Rectum	0.1 cc	101.30	100.50	0.84
	2 cc	74.62	73.96	0.80
Urinary bladder	0.1 cc	111.8	113.4	0.75
	2 cc	83.34	84.09	0.78
Sigmoid Colon	0.1 cc	92.13	94.27	0.72
	2 cc	61.15	63.73	0.44

The mean VAS scores for pain were 5.3, 4.8 and 4.5 for the first, the second and the third fractions of ICBT, respectively, in the CS group while it was 1.3 in the SA group.

## Discussion

As per the latest report of the Hospital Based Cancer Registries, 2021, released by ICMR for the year 2020, cervical cancer remains the second most common gynaecological cancer after breast cancer. The most common age group diagnosed with cervical cancer, according to this report is 45 to 55 years [21]. In this study, the most common age group of patients considering both the groups (SA and CS) was 50 to 60 years.

Squamous cell carcinoma was the predominant histopathology in our study (91%) which is in accordance with the 89.5% incidence of cervical cancer in India [21].

The most common stage of the disease at presentation was stage IIB, closely followed by stage IIIB [21].

In this study, we have collected data of 168 ICBT applications which is more in number than previous studies (138 applications in Sharma et al., 80 applications in Bana et al.) [22,23].

The mean point A dose in the left side (A2) was 99.53 % (6.96 Gy) in the SA group and 99.63% (6.97 Gy) in the CS group with a p-value of 0.77. In Bana et al., the average dose to point A2 was 5.75 Gy and 5.97 Gy respectively with a p-value of 0.64. The mean point A dose in the right side (A1) was 99.75 % (6.98 Gy) in SA group and 99.59% (6.97 Gy) in CS group with a p-value of 0.68. In Bana et al., the average dose to point A1 was 5.69 Gy and 5.92 Gy respectively with a p-value of 0.32 [23].

The mean point B dose in the left side was 29.98 % (2.09 Gy) in SA group and 27.87 % (1.95 Gy) in the CS group with a p-value of 0.25 (percentages are as % of point A dose). In Sharma et al., the mean dose to Point B in the left side was 1.89 Gy and 1.82 Gy, respectively, with a p-value of 0.01. The mean dose to Point B in the right side was 30.02 % (2.10 Gy) in SA group and 28.23% (1.98 Gy) in CS group with a p-value of 0.36. In Sharma et al., the mean dose to Point B in the right side was 1.91 Gy and 1.85 Gy respectively with a p-value of 0.07 [22]. In our study, dose coverage of Point B was found to be more than that.

The article "High-Dose-Rate Intracavitary Brachytherapy Under Conscious Sedation a Viable Practical Alternative to Spinal Anaesthesia in Carcinoma Cervix: A Retrospective Study in a Tertiary Care Centre in Eastern India" was published in 2021. Journal: Cureus.

The mean point P dose in the left side was 20.37 % (1.42 Gy) in SA group and 20.18% (1.41 Gy) in CS group with a p-value of 0.50. The mean point P dose in the right side was 20.26 % (1.42 Gy) in SA group and 20.45% (1.43 Gy) in CS group with a p-value of 0.54.

In our study, bladder D2 cc in SA and CS groups were 83.34% (5.83 Gy) and 84.09% (5.88 Gy), respectively (percentages are as % of point A dose). Similarly, D0.1 cc for bladder were 111.8% (7.82 Gy) in SA group and 113.4% (7.93 Gy) in the CS group. The above data suggests that the absolute values of bladder D2 cc and D0.1 cc were marginally lower in the SA group as compared to CS group but were not statistically significant (p-values 0.78 and 0.75 respectively). In Sharma et al., the mean dose to the bladder point was 5.03 Gy in anaesthesia group and 4.9 Gy in non-anaesthesia group respectively with a p-value of 0.6. [22] According to Bana et al., the maximum bladder dose in anaesthesia group ranges from 27.5% to 114.7% and in conscious sedation group, from 21.2% to 111% with a p-value of 0.04 which was significant. But the mean bladder doses were comparable in both the groups with a p-value of 0.13 which is similar to our study [23].

We found that rectum D2 cc in the SA and the CS groups were 74.62% (5.22 Gy) and 73.96% (5.17 Gy), respectively. Similarly, D0.1 cc for rectum were 101.3% (7.09 Gy) in SA group and 100.5% (7.03 Gy) in CS group. The above data suggests that the absolute values of bladder D2 cc and D0.1 cc were marginally higher in the SA group as compared to the CS group but were not statistically significant (p values 0.80 and 0.84 respectively). In Sharma et al., the mean dose to rectal point was 5.09 Gy in the anaesthesia group and 4.49 Gy in non-anaesthesia group respectively with p-value of 0.01, which was an unexpected finding, and they did not suggest any specific reason for this [20]. According to Bana et al., the maximum rectum dose in the anaesthesia group ranges from 26.2% to 90.4% and in the conscious sedation group, from 25.5% to 90% with a p-value of 0.054. Also, they found that mean rectum doses were comparable in both the groups with a p-value of 0.126 which is similar to our study [23].

Sigmoid D2 cc in SA and CS groups were 61.15% (4.28 Gy) and 63.73% (4.46 Gy), respectively. Similarly, D0.1 cc for sigmoid were 92.13% (6.45 Gy) in SA group and 94.27% (6.59 Gy) in CS group. The above data suggests that the absolute values of sigmoid D2 cc and D0.1 cc were marginally lower in the SA group as compared to CS group but were not statistically significant (p values 0.44 and 0.72 respectively).

The article "High-Dose-Rate Intracavitary Brachytherapy Under Conscious Sedation a Viable Practical Alternative to Spinal Anaesthesia in Carcinoma Cervix: A Retrospective Study in a Tertiary Care Centre in Eastern India" was published in 2021. Journal: Cureus.

This study shows there was no statistically significant difference, between the SA and the CS groups, in terms of dose to critical organs as well as dose to points A, B and P. The study by Anker et al. also revealed that anaesthesia had no role in terms of decreasing organ at risk dose and increasing pelvic wall dose [24].

The assessment of pain using VAS scores revealed that moderate pain was associated with ICBT under CS. It was also noted that the mean VAS scores gradually decreased with subsequent fractions of ICBT procedures. This may be attributed to the decreased burden of the disease or to the better knowledge of anatomy from the previous experience of the radiation oncologist.

As per ABS guidelines, there is no specific anaesthesia/sedation/analgesia recommendation for ICBT. So, we would like to suggest ICBT procedure under conscious sedation as a viable practice as it carries with itself a bunch of advantages. It can be done without specialist anaesthesia service, with lesser complications and on a day-care basis which in turn reduces hospital stay and bed occupancy. Additionally, the ease of induction of conscious sedation makes the procedure less time-consuming. So greater number of patient turnover can be achieved in a high-volume centre.

The number of plans evaluated were higher in comparison to earlier similar studies. Also, CT simulation and volumetric contouring of organs at risk (OAR) contouring were done. This provides a better input about the precise doses received by OARs as well as points A, B and P as compared to X-ray-based simulation. It also verifies the position of applicators as well. We also attempted to elaborate on urinary bladder, rectum and sigmoid colon dosages based on 0.1 cc and 2 cc doses, which was a novel attempt on analysis. In addition to points A and B, we also evaluated dose received by pelvic wall point (point P).

We feel that there are some caveats in our study. First, this is a retrospective study, so, a detailed prospective randomised study should be done. We have not analysed the clinical toxicity of organs at risk. Long-term follow-up is needed to correlate whether the dosimetric equivalence is being translated clinically.

## Conclusions

HDR-ICBT with CS is dosimetrically non-inferior to that with SA. The pain associated with the procedure in conscious sedation was also found to be moderate in nature. So ICBT with CS can be safely practised in centres with heavy burden of cervical cancer and lack of anaesthesia support. It can also be an acceptable choice for a patient who is not fit for anaesthesia. 
